# Aesthetic Effect of Autologous Fat Transplantation on Frontotemporal Depression Filling and Its Influence on SCL-90 and SES of Patients

This article has been retracted.

**DOI:** 10.1155/2022/3374780

**Published:** 2022-10-11

**Authors:** Dongjing Yin, Guoliang Shen

**Affiliations:** ^1^Department of Burns and Plastic Surgery, The First Affiliated Hospital of Soochow University, Suzhou 215006, Jiangsu, China; ^2^Department of Burns and Plastic Surgery, Affiliated Nantong Hospital 3 of Nantong University, Nantong 226000, Jiangsu, China

## Abstract

**Objectives:**

This study aimed to study the aesthetic effect of autologous fat transplantation in frontotemporal depression filling as well as the influence on the Symptom Checklist 90 (SCL-90) and the Rosenberg Self-Esteem Scale (SES) score of patients.

**Methods:**

A total of 100 patients with frontotemporal depression admitted to the outpatient department of burn and plastic surgery in our hospital were selected as the observation group, and all of them received autologous fat transplantation. The filling effect of patients in the observation group was discussed. Simultaneously, 50 volunteers were selected as the control group to compare the SCL-90 and SES scores of the observation group and the control group.

**Result:**

① A total of 100 patients with frontotemporal depression were treated with autologous fat transplantation, and the secondary autologous fat transplantation rate was 10%; two cases of fat absorption occurred during the 12-month follow-up after surgery; on the 7^th^ day, 6 months, and 12 months after the operation, the satisfaction rate of the patients who visited the doctor was 96.00%, 97%, and 92.00%; the satisfaction rate of the plastic surgeon was 94.00%, 96%, and 90.00%; the satisfaction rate of the third party was 96.00%, 98%, and 92.00%. ② The preoperative scores of somatization, obsessive-compulsive, interpersonal sensitivity, depression, anxiety, hostility, terror, paranoia, and psychotic factor scores in the observation group were higher than those in the control group (*P* < 0.05). The scores of somatization, obsessive-compulsive, interpersonal sensitivity, depression, anxiety, hostility, terror, paranoia, and psychotic factor scores in the observation group at 6 months after the operation were lower than those before operation (*P* < 0.05). The preoperative SES score of the observation group (28.51 ± 9.81) was significantly lower than that of the control group (32.47 ± 5.39) (*P* < 0.05). The SES score (34.17 ± 9.81) in the observation group at 6 months after the operation was significantly higher than that before the operation (*P* < 0.05).

**Conclusion:**

The aesthetic effect of autologous fat transplantation in frontotemporal depression filling is good and safe. Simultaneously, it can improve the mental health and self-esteem of patients and has high clinical value.

## 1. Introduction

With the increase in age, the lack of relaxation of soft tissues will lead to depression and deformity of the face. Once it seriously affects the appearance of the face, it is easy to give people a feeling of haggardness and sadness. More and more people have begun to pursue a kind of delicate and harmonious facial contour, and the main purpose is to make themselves look more beautiful and younger and meet their psychological needs for life, work, marriage, and love [1]. At present, in clinical practice, the materials for improving frontotemporal depression mainly include artificial materials and autologous materials, which are widely applied to the filling of frontal and temporal lobe depressions and have obvious aesthetic effects. However, compared with artificial materials, autologous materials have the significant advantages of low cost, no rejection, low infection incidence, and long effective period [2]. However, it has been found in clinical practice that the psychological state and self-esteem of plastic surgery patients are different from those of the general population due to the long-term effect of the disease [3]. In this study, autologous fat transplantation was applied in frontotemporal depression filling and achieved satisfactory aesthetic results. Simultaneously, the psychological status and self-esteem of patients were analyzed, and the report is as follows.

## 2. Materials and Methods

### 2.1. Research Objects

A total of 100 patients with frontotemporal depression who were admitted to the outpatient department of burn and plastic surgery in our hospital from January 2020 to August 2021 were selected as the observation group, and all received autologous fat transplantation. In the observation group, there were 14 males and 86 females; their age ranged from 24 to 66 years, with an average of (47.15 ± 3.37) years; there were 25 cases of simple frontal depression, 28 cases of simple temporal depression, and 47 cases of frontotemporal depression. Inclusion criteria were as follows: (1) meet the diagnostic criteria for congenital or aging frontotemporal depression and be diagnosed by a physician (fatty tissues and muscular tissues in the temporal part or frontal part are sunken due to atrophy, manifested as narrowing and prominence of the frontal part, forming the shape of upper small and lower wide or the lower limit of the frontal part, thus giving the impression of aging and fatigue); (2) there are no contraindications to surgery in the preoperative blood routine, coagulation function, blood sugar, and infection index tests; (3) age 24–66 years old, with complete case data available; (4) no cardiovascular disorder; (5) patients without AIDS, syphilis, hepatitis, and other infectious diseases; (6) all aware of the risks of surgery and signed the consent form for surgery. Exclusion criteria were as follows: (1) patients with mental disorders; (2) patients with insufficient blood supply or blood dysfunction in the surgical area; (3) patients who have previously injected substances such as fat and hyaluronic acid into the frontotemporal region; (4) patients with previous frontotemporal trauma, or skin damage, and body surface mass in the surgical area; (5) patients with contraindications for surgery; (6) women who are trying to conceive, breastfeeding, or pregnant. Simultaneously, 50 healthy volunteers with full frontotemporal were selected as the control group, and among them, there were 6 males and 44 females, aged from 24 to 64 years old, with an average of (47.18 ± 3.45) years. The general data (gender and age) of the two groups were similar (*P* > 0.05) and were comparable.

### 2.2. Methods

#### 2.2.1. Preoperative Preparation

After admission, the patient was diagnosed with frontotemporal depression and was informed of the surgical risk, then, the patient signed the surgical consent form, and the preoperative and postoperative photographs of the patient's surgical area were recorded. We carefully mark the concave range to roughly define the amount of fat to be filled; the liposuction site is selected from the inner thigh, and the liposuction area on one or both inner thighs is marked according to the amount of fat to be filled.

#### 2.2.2. Autologous Fat Extraction

Tumescent anesthesia was performed in the marked fat donor area, and a tumescent solution was made with 0.04% lidocaine +1 : 1 million epinephrine. We make an incision of about 4 cm on the outer upper side of the thigh, inject tumescent fluid with a water injection needle, 250 –300 ml of the unilateral thigh, evenly cover, place a water injection liposuction tube with a diameter of 4 cm in the incision, and connect a body-jet hydrodynamic-assisted liposuction system device (Human Med Company, Germany); the preoperative estimated fat was extracted by round-trip fan suction, and about 0.6 cm of subcutaneous fat was retained. A sufficient amount was extracted and placed in a syringe, the subcutaneous fluid was squeezed out, and the incision was sutured.

#### 2.2.3. Fat Purification

The extracted fat cells are placed in a larger container, the larger fat block is appropriately cut off, and the fat particles are purified by centrifugation. Specific operation method: after proper standing, we remove the impurities in the lower layer of fat particles, put the 10 ml syringe with the inner core removed into it, and put the centrifugal sleeve into the centrifuge; the centrifugation speed is 1000 rpm, and the centrifugation time is 5 minutes. The fat syringe was taken out from the centrifuge cannula, and the intact fat particles in the middle layer were taken and transferred to a 1 ml screw-capped syringe for later use.

#### 2.2.4. Fat Filling

In the temporal area, the inner edge of the intersection of the bilateral preauricular hairline and the temporal line was selected as the needle insertion point, and the forehead injection needle injection site was selected in the middle and two sides of the forehead hairline within 1 cm. The fat grafting area was anesthetized with 0.04% lidocaine from the distal end to the proximal end for local tumescent anesthesia; the prepared 1 ml of blunt fat was injected with 18 G blunt pressure into the concave site in fan-shaped, multitunnel, and cross-shaped uniform pressure to avoid agglomeration into clumps. We pay attention to the color and tension of the skin during injection to prevent damage to blood vessels and fat embolism; considering fat absorption, the amount of fat filling is about 20% greater than the volume of the depression. After surgery, the liposuction incision was sutured, and sterile dressings were used for pressure dressing; the liposuction area was compressed with elastic bandages for 3 d, and plastic leg pants were worn for at least 1 month; antibiotics were used for anti-infection after surgery for 5–7 days. The sutures are removed from the incision on the donor site; the injection point of fat filling should avoid touching water within 7 days after the operation. The fat grafting area should not be rubbed and pressed within 1 month after the operation, and spicy foods such as spicy and seafood should be contraindicated within 1 to 3 months after the operation. High collagen food was eaten; follow-up was performed 7 days, 6, and 12 months after surgery, and the amount of fat transplantation, satisfaction, and complications was counted.

#### 2.2.5. Follow-Up

All patients were followed up for one year after the operation, and their recovery was known by telephone or outpatient service every month, and the occurrence of adverse reactions was observed.

### 2.3. Fat Survival Rate and Satisfaction Assessment

Fat survival rate = (measurement of frontotemporal volume at 6 months follow-up preoperative frontotemporal volume)/injected fat volume^*∗*^100%. The number of fat transplants during the 12-month follow-up period was recorded, and satisfaction was assessed [4]. 7 d after the operation, 6 months after the operation, and 12 months after the operation, the satisfaction evaluation of the patients in the observation group was evaluated by patients themselves, plastic surgeons, and a third person not related to this study. The evaluation was rated on a scale of 1–5, with 5 points indicating very satisfactory and 1 point indicating completely unsatisfactory. The satisfaction rate = (5 points cases +4 points cases)/total cases ×100%.

### 2.4. Symptom Assessment

Self-report symptom inventory Symptom Checklist 90 (SCL-90) evaluation [5]: the patients of control group admitted on the 1st day and the patients of observation group admitted on the 1st day and 6 months after the operation, filled out the SCL-90 questionnaire under the unified guidance of professionals, and the questionnaire involved various mental health problems, which were summarized into somatization, obsessive-compulsive, interpersonal sensitivity, depression, anxiety, hostility, terror, paranoia, and psychotic factors. Each item of SCL-90 was divided into 1–5 points according to its severity. The higher the score, the more serious the symptoms. If the total score of SCL-90 was greater than 160, the number of positive items was more than 43, or if the average score of any major item was more than 2, then the patient could be considered to have positive symptoms.

### 2.5. Self-Esteem Assessment

Rosenberg Self-Esteem Scale (SES) evaluation [6]: The patients of control group admitted on the 1st day and the patients of observation group admitted on the 1st day and 6 months after the operation,filled out the SES questionnaire under the unified guidance of professionals. The questionnaire included 10 items. Each item was scored as “very agree,” “agree,” “disagree,” and “strongly disagree” with 1–4 points, with the total score ranging from 10 to 40 points. A higher SES score indicates higher self-esteem.

### 2.6. Evaluation of Complications

Complications, including infection, fat liquefaction, and nodules, were recorded during the postoperative follow-up in both groups.

### 2.7. Statistical Analysis

All data were processed by SPSS 23.0 statistical software package, measurement data were expressed as mean ± standard deviation ($\bar{x}$ ±S), using the *t*-test; enumeration data were described by the pass rate/composition ratio, using the *χ*^2^ test, with *P* < 0.05 as the statistical difference study meaning.

## 3. Results

### 3.1. Analysis of Fat Transplantation Survival Rate and Satisfaction Results

During the 6 months follow-up after the operation, the fat survival rate was higher (69.84 ± 4.83) %; the satisfaction rate of those seeking medical treatment on the 7^th^ day, 6 months, and 12 months after the operation was 96.00%, 97%, and 92.00%; the satisfaction rate of plastic surgeons was 94.00%, 96%, and 90.00%; the third-party satisfaction rate was 96.00%, 98%, and 92.00%, as shown in Tables 1–3.

### 3.2. Comparison of SCL-90 and SES Scores between the Observation Group and the Control Group

The preoperative scores of somatization, obsessive-compulsive, interpersonal sensitivity, depression, anxiety, hostility, terror, paranoia, and psychotic factor scores in the observation group were higher than those in the control group (*P* < 0.05). The scores of somatization, obsessive-compulsive, interpersonal sensitivity, depression, anxiety, hostility, terror, paranoia, and psychotic factor scores in the observation group at 6 months after the operation were lower than those before the operation (*P* < 0.05) (see Table 4). The preoperative SES score of the observation group (28.51 ± 9.81) was significantly lower than that of the control group (32.47 ± 5.39) (*P* < 0.05). The SES score of the observation group 6 months after surgery (34.17 ± 9.81) was significantly higher than that of the preoperative (34.17 ± 9.81) (*P* < 0.05).

### 3.3. Complications during Follow-Up

A total of 100 patients with frontotemporal depression were treated with autologous fat transplantation, and most of the patients were accompanied by local redness and swelling 7 days after the operation. The 10 patients who sought medical treatment showed no obvious improvement. After communication and consultation, second autologous fat transplantation was performed 6 months later. The secondary transplantation rate was 10%, and the effect was satisfactory. During the 12-month follow-up period, 2 patients had fat absorption, and no complications occurred such as infection, subcutaneous mass, and uneven skin.

## 4. Discussion

When facial aging develops to a certain extent, there will be depression, relaxation, and wrinkles in the facial skin and soft tissue. At present, clinicians can repair the depression contour of a patient using a filling technique, in which the autologous fat filling technique has been widely used [7]. Autologous fat filling is to absorb excess subcutaneous fat cells from certain parts of the human body, purify sucked fat, and then select complete autologous fat cells by injection and then transplant them to the site that needs fat filling [8, 9]. Autologous fat, which is derived from the subject itself, has the advantages of no immunologic rejection, wound, and long use time, and meanwhile, compared with artificial materials, autologous materials impose a less economic burden on the patient. However, because the blood circulation of fat cells can be damaged after inhalation and a series of treatments, some fat cells are difficult to survive and can cause rapid necrosisafter transplantation. Long-term clinical observations have found that the survival rate of fat cells after transplantation is between 10% and 80%, and most patients require secondary autologous fat transplantation due to a lack of conscious improvement [10, 11]. In this study, 100 patients with frontotemporal depression were treated with autologous fat transplantation. After 6 months of follow-up, the fat survival rate was (69.84 ± 4.83) %, which was relatively high, but 10 patients (10%) were not significantly improved. The key to fat filling is to improve the fat survival rate, and the fat survival rate is mainly related to methods such as fat extraction and purification. The most commonly used liposuction method in the clinic is the negative pressure liposuction method. The principle of negative pressure liposuction is to suck out subcutaneous fat by using the negative pressure generated by the machine, which has the advantages of convenient operation and short operation time. At 50 kPa, with the increase of pressure, the surgical injury and fat damage will be more serious, which will reduce the fat survival rate, and the rate of secondary fat transplantation will be higher [12, 13]. Simultaneously, studies have shown [14] that when the negative pressure of liposuction is less than 50 kPa, there is no difference in the damage of fat cells under different pressures. In this study, the German Body-Jet hydrodynamic system is used to have a closed fat recovery mechanism, and while directly filtering and separating the extracted fat, it can also remove suctioned fibrous connective tissue. After the method is used, the purity of sucked axillary lower layer fat particles is higher, and meanwhile, fat can be stored in a closed sterile environment in each link of the surgical operation, so that the separation time of fat particles can be reduced, and the infection rate and necrosis rate are reduced, the fat survival rate is further improved, and finally, a satisfactory aesthetic effect is achieved. In addition, some studies believe that the application of autologous fat transplantation has certain risks. Common postoperative complications include induration, fat absorption, subcutaneous mass, and infection, but they can be controlled by standard surgical operations [15]. At present, the safety factor of autologous fat transplantation is getting higher and higher, and the operation technology and the experience of operators are becoming more and more mature. In this study, only 2 cases out of 100 patients with frontotemporal depression were complicated by liposuction, and this conclusion is consistent with the above viewpoint and indicates that autologous fat transplantation is a safer method for filling frontotemporal inhibition. The reasons were analyzed: (1) all the autologous fat transplantation was performed by experienced senior physicians, and the hydrodynamic liposuction method was used to reduce the complications of autologous fat transplantation to avoid damage to fat cells; (2) a 2.5 mm liposuction tube is used during liposuction to avoid the liposuction tube being too thin to damage the integrity of fat particles and reduce the risk of fat absorption and uneven skin surface; (3) we use a blunt needle to inject fat to fill and inject evenly in the form of a fan-shaped, multitunnel, and cross-shaped depression in order to avoid agglomeration into agglomerates; (4) we pay attention to the color and tension of the skin during injection to prevent damage to blood vessels and fat embolism. In addition, in order to prevent postoperative infection and reduce the survival rate of adipose cells, strict aseptic operation should be performed during the operation, and antibiotics should be used to resist infection within 5–7 days after the operation.

According to the survey, the aging of facial depression not only affects people's physical feelings but also affects people's mental health to a certain extent, resulting in some people's lack of self-confidence and fear of participating in social activities [16]. In this study, the preoperative somatization, obsessive-compulsive, interpersonal sensitivity, depression, anxiety, hostility, terror, paranoia, and psychotic factor scores in the observation group were higher than those in the control group (*P* < 0.05). The preoperative SES score of the observation group was (28.51 ± 9.81) points, which was significantly lower than that of the control group (32.47 ± 5.39) (*P* < 0.05), and the results show that frontotemporal depression filling patients have negative emotions such as anxiety and depression in terms of mental health, accompanied by somatic symptoms and personality paranoia, especially expressed as interpersonal sensitivity and compulsion. In terms of self-esteem levels, it is manifested as disapproval and unacceptance of self, and an obvious inferiority complex appears. The results suggest that medical workers need time and energy to solve the psychological problems of such patients while doing routine medical care work [17, 18]. In this study, the scores of somatization, obsessive-compulsive, interpersonal sensitivity, depression, anxiety, hostility, terror, paranoia, and psychotic factor scores in the observation group 6 months after operation were lower than those before operation (*P* < 0.05). The SES score of the observation group 6 months after the operation was significantly higher than that before the operation (*P* < 0.05), and the results showed that the psychological status and self-esteem of the patients treated with autologous fat transplantation for frontotemporal depression were significantly improved after surgery. Autologous fat filling can greatly improve the facial aesthetics of patients, which can affect the psychological state and self-esteem of patients to some extent [19].

In conclusion, autologous fat transplantation has a good and safe aesthetic effect in frontotemporal depression filling and can improve the mental health and self-esteem of medical patients, which has high clinical value. However, the authors believe that this study still has limitations, such as a single study sample and a short follow-up time. In particular, the aesthetic effects of patients with different levels of fat extraction and purification and different degrees of frontotemporal depression have not been analyzed. The research conclusions are worthy of further verification.

## Figures and Tables

**Table 1:** Satisfaction evaluation of patients, plastic surgeons, and third parties on the 7^th^ day after the operation.

Indexes	Patients					Plastic surgeons					3rd party (third party not related to this study)				
Score	5	4	3	2	1	5	4	3	2	1	5	4	3	2	1
Number of cases	86	10	0	4	0	84	10	4	2	0	88	8	4	0	0
Percentage	86.00	10.00	0	4.00	0	84.00	10.00	4.00	2.00	0	88.00	8.00	4.00	0	0
Satisfaction rate %	96.00					94.00					96.00				

**Table 2:** Satisfaction evaluation of patients, plastic surgeons, and third parties 6 months after surgery.

Indexes	Patients					Plastic surgeons					3^rd^ party (third party not related to this study)				
Score	5	4	3	2	1	5	4	3	2	1	5	4	3	2	1
Number of cases	86	11	0	3	0	83	13	3	1	0	88	10	2	0	0
Percentage	86.00	11.00	0	3.00	0	83.00	13.00	3.00	1.00	0	88.00	10.00	2.00	0	0
Satisfaction rate %	97.00					96.00					98.00				

**Table 3:** Satisfaction evaluation of patients, plastic surgeons, and third parties 12 months after surgery.

Indexes	Patients					Plastic surgeons					3^rd^ party (third party not related to this study)				
Score	5	4	3	2	1	5	4	3	2	1	5	4	3	2	1
Number of cases	86	6	6	2	0	84	6	6	2	2	82	10	4	4	0
Percentage	86.00	6.00	6.00	2.00	0	84.00	6.00	6.00	2.00	2.00	82.00	10.00	4.00	4.00	0
Satisfaction rate %	92.00					90.00					92.00				

**Table 4:** Comparison of SCL-90 scores between the observation group and the control group ($\bar{x}$ ± *s*, points).

Group	Somatization	Obsessive-compulsive	Interpersonal sensitivity	Depression	Anxiety	Hostility	Terror	Paranoia	Psychotic
Control group (*n* = 50)	1.36 ± 0.47	1.61 ± 0.56	1.59 ± 0.60	1.49 ± 0.58	1.38 ± 0.42	1.45 ± 0.44	1.22 ± 0.40	1.42 ± 0.56	1.28 ± 0.41
Observation group (*n* = 100)									
Before surgery	1.51 ± 0.55^a^	1.94 ± 0.84^a^	1.93 ± 0.64^a^	1.69 ± 0.61^a^	1.53 ± 0.52^a^	1.39 ± 0.33^a^	1.22 ± 0.39^a^	1.59 ± 0.50^a^	1.44 ± 0.48^a^
6 months after surgery	1.35 ± 0.48^b^	1.59 ± 0.79^b^	1.41 ± 0.62^b^	1.50 ± 0.59^b^	1.37 ± 0.51^b^	1.40 ± 0.46^b^	1.21 ± 0.37^b^	1.41 ± 0.52^b^	1.26 ± 0.39^b^
*t* value of preoperative and control group	3.341	4.172	3.714	3.165	3.914	1.064	0.861	4.028	3.467
*P* value of preoperative and control group	0.033	0.027	0.029	0.037	0.031	0.079	0.144	0.019	0.032
*t* value of 6 month postoperative and preoperative	3.247	4.039	3.451	3.046	3.461	1.174	0.797	3.972	3.243
*P* value of 6 month postoperative and preoperative	0.035	0.025	0.030	0.038	0.034	0.516	0.115	0.026	0.036

*Note.* ^a^ *P* < 0.05, compared with the control group; ^b^*P* < 0.05, compared with the observation group before the operation.

## Data Availability

The data used and/or analyzed during the current study are available from the corresponding author.
